# Effects of natural aging and gender on pro-inflammatory markers

**DOI:** 10.1590/1414-431X20198392

**Published:** 2019-08-12

**Authors:** J.C. Milan-Mattos, F.F. Anibal, N.M. Perseguini, V. Minatel, P. Rehder-Santos, C.A. Castro, F.A. Vasilceac, S.M. Mattiello, L.H. Faccioli, A.M. Catai

**Affiliations:** 1 Laboratório de Fisioterapia Cardiovascular, Núcleo de Pesquisas em Exercício Físico, Departamento de Fisioterapia, Universidade Federal de São Carlos, São Carlos, SP, Brasil; 2 Departamento de Morfologia e Patologia, Universidade Federal de São Carlos, São Carlos, SP, Brasil; 3 Laboratório de Função Articular, Departamento de Fisioterapia, Universidade Federal de São Carlos, São Carlos, SP, Brasil; 4 Departamento de Análises Clínicas, Toxicológicas e Bromatológicas, Faculdade de Ciências Farmacêuticas de Ribeirão Preto, Universidade de São Paulo, Ribeirão Preto, SP, Brasil

**Keywords:** Natural aging, Inflammaging, Immune system, hsCRP, IL-6

## Abstract

The term inflammaging is now widely used to designate the inflammatory process of natural aging. During this process, cytokine balance is altered, presumably due to the loss of homeostasis, thus contributing to a greater predisposition to disease and exacerbation of chronic diseases. The aim of the study was to analyze the relationship between pro-inflammatory markers and age in the natural aging process of healthy individuals. One hundred and ten subjects were divided into 5 groups according to age (22 subjects/group). Interleukin-6 (IL-6) and tumor necrosis factor α (TNF-α) were quantified using the ELISA method. High-sensitivity C-reactive protein (hsCRP) was analyzed by turbidimetry according to laboratory procedures. The main findings of this study were: a positive correlation between hsCRP and IL-6 as a function of age (110 subjects); women showed stronger correlations; the 51–60 age group had the highest values for hsCRP and IL-6; women presented higher values for hsCRP in the 51–60 age group and higher values for IL-6 in the 61–70 age group; and men showed higher values in the 51–60 age group for hsCRP and IL-6. In conclusion, the natural aging process increased IL-6 and hsCRP levels, which is consistent with the inflammaging theory; however, women presented stronger correlations compared to men (IL-6 and hsCRP) and the 51–60 age range seems to be a key point for these increases. These findings are important because they indicate that early preventive measures may minimize the increase in these inflammatory markers in natural human aging.

## Introduction

The immune system is the mechanism that enables homeostasis throughout our lifetime. From birth, this system initiates modifications that allow the functional maturation of its effectors. Over the years, these changes begin to show decreased activity and weakened immediate response, especially in innate immunity, thus contributing to systemic and cardiovascular changes, which may or may not impair the individual (1).

With the advances in medical care and sanitation, there has been a tremendous increase in human life expectancy, with population aging now becoming one of the greatest challenges to contemporary public health. This phenomenon occurred initially in developed countries, but more recently it has risen more sharply in developing countries (1).

In this context, the term “inflammaging” has become widely used to describe the characteristic inflammatory process of aging. Inflammaging is characterized by a subclinical, low-grade, chronic systemic pro-inflammatory state (2,3). During this process, the balance of cytokines in the body undergoes changes, probably due to loss of homeostasis, which contributes to a greater predisposition to illness and worsening of chronic diseases such as hypertension and diabetes. Thus, inflammaging seems to be associated with increased morbidity and mortality in the elderly (4,5).

This low-grade, chronic systemic pro-inflammatory state consists of elevated levels of pro-inflammatory cytokines, such as interleukin-1 (IL-1), interleukin-6 (IL-6), and tumor necrosis factor α (TNF-α), and appears to be involved in the pathogenesis of various age-related diseases. Another component widely used in clinical practice as a marker of inflammaging is C-reactive protein (CRP), which is produced in response to IL-6 and is also a robust predictor of risk for cardiovascular disease (6,7).

The pro-inflammatory cytokines IL-6 and TNF-α are commonly studied, and there is consensus about the increased concentrations in elderly subjects for both IL-6 (8,9) and TNF-α (8,10–12). IL-6 is considered the cytokine of gerontologists (13). Combined with TNF-α, it induces CRP production, which is useful as an inflammatory marker in the aging process and most commonly used in clinical practice (6,13).

A central problem in studies on aging of the immune system is the difficulty in obtaining data from very healthy elderly individuals in order to identify the physiological changes in the natural aging process without the presence of disease. Also, there are few studies that evaluate the changes in the immune system separately by gender (14,15). Therefore, the aim of this study was to evaluate the levels of the inflammatory markers IL-6, TNF-α, and high-sensitivity CRP (hsCRP) in healthy men and women of different age groups, and to analyze the relationship between these pro-inflammatory markers and age in the natural aging process.

## Material and Methods

### Participants

One hundred and ten individuals were assigned to 5 groups according to age: 21–30, 31–40, 41–50, 51–60, and 61–70 years with 22 subjects in each group (11 men and 11 women). Anthropometric measurements including weight (in kg) and height (to the nearest cm) were recorded for all participants. Body mass index (BMI) was calculated using the formula: weight (kg)/height^2^ (m^2^).

The exclusion criteria were as follows: BMI≥30 kg/m^2^, alcohol or smoking habit, diabetes, hypertension, use of illicit drugs or medications that could affect the responses of the variables, and for women, use of contraceptives or hormone replacement therapy. In addition, individuals with a history of inflammation and hsCRP serum values suggestive of acute inflammation were excluded, i.e., above the normal upper limit: 3.0 mg/L (16).

The study participants were informed about the procedures and methods to be used in the study. After agreeing to take part in the study, the participants read and signed an informed consent form. This study followed the Declaration of Helsinki guidelines and was approved by the Human Research Ethics Committee of the Federal University of São Carlos (protocol #328 472).

### Clinical evaluation

The participants underwent clinical and functional assessment including anamnesis to identify personal characteristics, lifestyle habits, physical activity, use of medication, and presence of disease or known risk factor. This assessment was used to evaluate the criteria for inclusion and exclusion from the study.

### Cardiopulmonary exercise testing

Participants underwent a cardiopulmonary exercise test on a treadmill (Master ATL, Inbramed, Brazil) for the aerobic functional classification. The incremental protocol was used and the test was interrupted in the presence of signs or symptoms of fatigue reported by the participant, as described by Neves et al. (17). The ventilatory and metabolic parameters were captured and recorded breath-by-breath through a cardiopulmonary exercise system (CPX/D, Medical Graphics, USA). Peak VO_2_ was defined as the maximum oxygen consumption (VO_2_) observed in the final 30 seconds of exercise and was considered in absolute values (mL/min) and relative values corrected for body weight (mL·kg^-1^·min^-1^). Electrocardiography was performed continuously throughout the test using an electrocardiograph (WinCardio, Micromed Biotechnology Ltda., Brazil) and blood pressure was measured using the auscultatory method. Perceived exertion was assessed every 2 min using the CR10-Borg Scale (18).

### Blood collection

Blood was collected in the morning after a 12-hour fast. Venous blood was collected by puncture of the antecubital vein in vacuum tubes without anticoagulant by experienced personnel in a specialized laboratory. One part of the blood sample was used for total cholesterol, high-density lipoprotein (HDL), low-density lipoprotein (LDL), very-low-density lipoprotein (VLDL), triglycerides, glycemia, and hsCRP analysis, and the other part was centrifuged at 1008 *g* for 10 min to separate the serum. The supernatant was relocated to 2.0 mL microtubes and stored in a freezer at –80°C for subsequent analysis of the quantification of inflammatory cytokines levels. For women of reproductive age, blood sampling was performed between the 7th and 10th day of the menstrual cycle (follicular phase) to ensure that the collection was not performed during the menstruation period.

### hsCRP measurements

The turbidimetry method was used for hsCRP analysis according to laboratory procedures.

### Cytokine measurements

Cytokines were quantified in serum using the enzyme-linked immunosorbent assay (ELISA) method according to the manufacturer's instructions (OptEIA Set BD Biosciences, USA). The cytokines IL-6 and TNF-α were detected using capture antibody (anti-human TNF-α and IL-6), standard cytokine, and detection antibody (biotinylated anti-human TNF-α and IL-6) and were amplified with avidin-peroxidase (streptavidin-horseradish peroxidase conjugate). As substrate, tetramethylbenzidine (TMB) was used and the reaction was blocked by adding sulfuric acid (2NH_2_SO_4_). The reading of the samples was performed on a 450 nm filter and the sensitivity threshold of the ELISA with serum was specified according to the manufacturer's indications.

### Statistical analysis

SigmaPlot 11.0 software (Systat Software, Inc., USA) was used. The Shapiro-Wilk test was used to verify the normality of data distribution; the variables that showed non-normal distribution were transformed using logarithmic function. Data were analyzed using two-way analysis of variance (ANOVA). One-way ANOVA with Tukey's post-hoc test and Kruskal-Wallis ANOVA on ranks with Dunn's post-hoc test were used to analyze the participants' characteristics and biochemical variables. The Spearman correlation test was also used. The level of significance was P<0.05. To evaluate the influence of the biochemical variables (cholesterol, HDL, LDL, triglycerides, and glycemia) on the outcome variables (hsCRP, IL-6, and TNF-α) in each age group, multivariate linear regression was performed using the stepwise method.

## Results

The age and anthropometric characteristics of the 110 study participants, divided into age groups and divided by gender, were described by Catai et al. (19). There was no statistical difference for weight and height. As expected, there were differences for BMI, with higher values in the older groups compared to the younger groups. However, the 41–50 group showed higher values compared to 21–30 and 31–40 groups. When only women were compared, groups 41–50 and 61–70 had higher BMI values compared to the youngest group and 61–70 had higher values compared to 31–40. Peak VO_2_ was lower in 61–70 and 41–50 compared to 31–40 and it was lower in 61–70 compared to 21–30 and 41–50. For the men's comparison, peak VO_2_ was lower in 61–70 compared to 21–30, 31–40, and 41–50. For the women's peak VO_2_, 61–70 and 51–60 had lower values compared to 21–30 and 31–40, while 61–70 had lower values compared to 41–50.

Regarding the blood tests (means±SD), total cholesterol was higher in groups 41–50, 51–60, and 61–70 compared to the younger groups, while LDL showed higher values in 41–50, 51–60, and 61–70 compared to 21–30 and a higher value in 51–60 compared to 31–40. In addition, the triglycerides were higher in 51–60 and 61–70 compared to 21–30. The same occurred with VLDL. Glycemia showed a higher value in group 61–70 compared to 21–30. HDL showed no significant difference between groups (Table 1).

**Table 1.** Overall biochemical results according to age groups (in years) and according to sex and age groups.

Characteristics	21–30	31–40	41–50	51–60	61–70
110 volunteers (n=11M,11F/group)					
Total Chol (mg/dL)	156.68±28.91	190.91±35.82	200.73±32.84^*^	223.27±46.16^*^	211.76±41.48^*^
LDL (mg/dL)	82.91±27.09	103.50±27.64	122.32±30.53^*^	135.32±44.20^*+^	127.62±33.21^*^
HDL (mg/dL)	55.77±13.08	66.00±30.40	57.50±17.59	60.95±16.63	58.57±13.35
Triglycerides (mg/dL)	85.14±50.93	97.91±52.05	99.77±47.63	130.77±57.68^*^	123.43±47.91^*^
Glycemia (mg/dL)	87.54±4.96	89.14±6.51	91.82±8.92	93.23±6.72	95.90±8.02^*+^
Males (n=11M/group)					
Total Chol (mg/dL)	161.64±30.94	190.45±34.15	201.00±41.37	218.45±30.53^*^	204.64±26.30^*^
LDL (mg/dL)	89.91±29.22	111.82±28.31	131.64±35.12^*^	135.91±23.47^*^	125.64±19.82^*^
HDL (mg/dL)	50.54±13.84	53.27±10.78	46.82±6.65	55.09±13.15	52.00±11.54
Triglycerides (mg/dL)	100.27±69.41	122.73±53.57	107.91±43.58	132.82±52.48	129.82±56.69
Glycemia (mg/dL)	89.27±5.98	90.82±8.07	95.36±9.23	92.36±5.06	94.54±6.15
Females (n=11F/group)					
Total Chol (mg/dL)	151.73±27.26	191.36±39.08	200.45±23.51^*^	228.09±59.08^*^	219.60±54.07^*^
LDL (mg/dL)	75.91±24.08	95.18±25.50	113.00±23.09	134.73±59.59^*^	129.80±44.78^*^
HDL (mg/dL)	61.00±10.38	78.73±38.31	68.18±18.83	68.18±18.83	65.80±11.72
Triglycerides (mg/dL)	70.00±11.18	73.09±38.27	91.64±52.16	128.73±64.98	116.40±37.76
Glycemia (mg/dL)	85.82±3.06	87.45±4.20	88.27±7.35	94.09±8.21	97.40±9.80^*+#^

Data are reported as means±SD. Chol: cholesterol; LDL: low-density lipoprotein; HDL: high-density lipoprotein. *P<0.05 compared to 21–30; ^+^P<0.05 compared to 31–40; ^#^P<0.05 compared to 41–50 (one-way ANOVA with Tukey test post-hoc or Kruskal-Wallis one-way ANOVA on ranks with post-hoc Dunn's test).

In the division by gender, the men's group showed higher values for total cholesterol in 51–60 and 61–70 compared to 21–30. LDL was higher in 41–50, 51–60, and in 61–70 compared to 21–30. HDL, triglycerides, and glycemia showed no significant differences between age groups. For women, the 41–50, 51–60, and 61–70 groups presented higher values for total cholesterol when compared to 21–30. LDL was higher in 51–60 and 61–70 compared to 21–30. Glycemia was higher in 61–70 compared to 21–30, 31–40, and 41–50 (Table 1).

Additionally, the multivariate linear regression analysis showed that the biochemical variables did not influence the responses of the outcome variables (hsCRP, IL-6, and TNF-α) of this study in any of the groups.

Figure 1 presents the data for hsCRP and the relationship of hsCRP as a function of age in the studied age groups and divided by gender. The analysis showed that the 51–60 group had the highest hsCRP values compared to the other groups. There was no interaction between gender and group for hsCRP. However, there was a positive correlation with age in the 110 participants (r=0.369), men (r=0.286), and women (r=0.451).

**Figure 1.** High sensitivity C-reactive protein (hsCRP) of the 110 volunteers (**A**) and divided by gender (**B**). Data are reported as means±SD. *P<0.05 compared to all the other age groups (two-way analysis of variance). hsCRP as function of age of the 110 volunteers (**C**), men (**D**), and women (**E**). •: 21–30; ○: 31–40; ▾: 41–50; Δ: 51–60; ▪: 61–70. Spearman correlation coefficient (r).

The data related to TNF-α are shown in Figure 2. There was no significant difference between the studied groups. In addition, there was no correlation between this variable and age in any of the three analyses: 110 participants, male, and female. However, it was possible to identify a trend toward increased TNF-α levels as a function of age (Figure 2).

**Figure 2.** Tumor necrosis factor α (TNF-α) of the studied age groups of the 110 volunteers (**A**) and divided by gender, (**B**). Data are reported as means±SD. TNF-α as function of age of the 110 volunteers (**C**), men (**D**), and women (**E**). •: 21–30; ○: 31–40; ▾: 41–50; Δ: 51–60; ▪: 61–70.

Two-way ANOVA showed the effects of IL-6 on the groups. Men had higher values in the 51–60 age group compared to 21–30, 31–40, and 61–70. The women had higher values in 61–70 compared to 21–30 and 31–40. In addition, only the 51–60 age group showed effect of gender, with men presenting higher values of IL-6. However, there was a positive correlation with age in the analyses: 110 participants (r=0.399), male (r=0.303), and female (r=0.555) (Figure 3)

**Figure 3.** Interleukin 6 (IL-6) of the 110 volunteers (**A**) and divided by gender (**B**). Men: *P<0.05 compared to 21–30, 31–40, and 61–70; Women: ^+^P<0.05 compared to 21–30 and 31–40; ^±^statistical difference between men and women in 51-60 (two-way analysis of variance). Right panels: hsCRP as a function of age of the 110 volunteers (**C**), men (**D**), and women (**E**). •: G21–30; ○: G31–40; ▾: G41–50; Δ: G51–60; ▪: G61–70. Spearman correlation coefficient (r) and P<0.05.

## Discussion

In this study, the assessment of healthy individuals of different ages allowed us to analyze the influence of age and gender on the levels of hsCRP, IL-6, and TNF-α in a large group of healthy subjects. The main findings of this study were: 1) there was a positive correlation between hsCRP and IL-6 as a function of age in all data (110 participants); 2) when the participants were divided by gender, women showed stronger correlations than men; 3) in the analysis of all participants, the 51–60 age group had the highest values for hsCRP and IL-6; 4) women presented higher values for hsCRP in the 51–60 age group and higher values of IL-6 in the 61–70 age group; and 5) men showed higher values in the 51–60 age group for hsCRP and IL-6.

Although the older age groups had higher BMI values compared to the 21–30 age group, it is worth noting that these values are within normal limits and below the obesity cutoff (>30 kg/m^2^). It is well known that obesity is associated with increased inflammatory markers, particularly IL-6, since adipocytes are sources of IL-6 (20,21).

However, LDL cholesterol, total cholesterol, triglycerides, and glycemia increased with age, and these findings are consistent with the changes that occur in aging due to the changes in regulatory mechanisms (22,23).

As previously mentioned, multivariate linear regression analysis showed that data from the biochemical analysis did not influence the responses of the outcome variables of this study (hsCRP, IL-6, and TNF-α). The analysis of hsCRP plasma levels as a function of age indicated that hsCRP increased with age and that the 51–60 age group had the highest values compared to the other groups when all participants were analyzed; however, all of them had values within the normal range. In the analysis of IL-6, the results were similar, i.e., increased levels as a function of age. In the analysis according to gender, men had higher values in the 51–60 age group and women had higher values in the 61–70 age group.

The analysis of the TNF-α level did not demonstrate differences among the five groups, but it was possible to identify a trend toward increased levels of this inflammatory marker as a function of age and higher values in the 61–70 group. The fact that TNF-α, which is the precursor of IL-6 and consequently of CRP, did not change in the same way as the other markers could be explained by the ability of IL-6 to inhibit the production of TNF-α, which, contrary to expectations, results in maintenance levels of TNF (24,25). Furthermore, Goetzl et al. (15) suggest that TNF-α is difficult to detect in healthy subjects.

Several studies have aimed to investigate the levels of cytokines in natural aging; however, the results are contradictory because many are *in vitro* studies (26,27) and there is also the problem of distinguishing natural aging from pathological aging (11). Gonzalo-Calvo et al. (11) evaluated IL-6 and TNF-α levels in apparently healthy elderly (mean age 83 years, 55% female) and middle-aged subjects (18–40, mean age 26 years, 47% female) using the ELISA kit. The analysis of IL-6 did not identify differences between the groups. TNF-α was statistically higher in the elderly group compared to the middle-aged group. Our study is not in agreement with the study of Gonzalo-Calvo et al. (11) possibly because this study did not analyze the same number of men and women in each group or because the mean age of the elderly group was higher than the mean age of our sample.

Our findings were in agreement with those of Alvarez-Rodrigues et al. (10), who evaluated 73 healthy subjects divided into young (26.2±2.4), middle-aged (44.7±8.4), and elderly (70.6±7.9) groups with no history of inflammation. They reported a positive correlation between IL-6 and age (r=0.664), although the levels of IL-6 were significantly higher in the elderly group compared to the other groups. In the same study, the TNF-α level presented a positive correlation with age (0.368), and the elderly and middle-aged groups showed higher values compared to the young group. Our findings corroborated their study, indicating that there is a positive correlation between IL-6 and TNF-α plasma levels and age, as well as increased IL-6 in older age groups. Although we found no significant differences between the groups with respect to TNF-α, it is noteworthy that, in the study of Alvarez-Rodrigues et al. (10), the elderly group also had a higher mean age than our study.

Unlike the studies mentioned above, the present work excluded participants with abnormal hsCRP because they could have an undetectable subclinical infection or disease. In addition, the participants were divided into five groups with an equal number of men and women in each group, not allowing a high value of standard deviation for age.

The concern to equalize the number of men and women in all age groups occurred due to the fact that women are more susceptible to autoimmune diseases (28,29), although the reason for this is still not fully understood. In women, hormonal changes seem to play an important role in changes in levels of inflammatory markers. Several conditions can alter estrogen levels, including the use of medications (corticosteroids, oral contraceptives, and hormone replacement therapy), menstrual cycle, menopause, etc. Therefore, in this study, the use of oral contraceptives and hormone replacement therapy was an exclusion criterion. For all pre-menopausal female participants, blood sampling was always performed between the 7th and 10th days of the menstrual cycle, and for the post-menopausal women, the absence of menstruation for at least one year prior to collection was confirmed (28).

In the present study, the increase in IL-6 levels was more prominent in the 51–60 age group, where 10 of the 11 women were in menopause. The next age group had the higher value, with all of the women in menopause. Our study is in accordance with Cioffi et al. (30) who reported that women in menopause have higher levels of IL-6 compared to fertile women. Increased levels of IL-6 in postmenopausal women appear to be associated with estrogen deficiency, which leads to a greater response of the body's cells to these cytokines as a consequence of the increase in the number of cytokine receptors and cofactors that facilitate cytokine action (31). In addition, estrogen deprivation in this stage of life appears to be associated with other diseases that occur more in menopause, such as diabetes, atherosclerosis, and cardiovascular diseases (28,29).

With respect to IL-6 levels in men, the group 51–60 had the highest values. For this variable, men experienced high IL-6 serum levels before women. Bonafà et al. (14) evaluated 700 volunteers between the age of 60 and 110 years and divided them into three age groups. The authors found that women experience higher IL-6 levels later in life compared to men and that the age-related increase in IL-6 in women is independent of genetic factors. These findings agree with the study of Franceschi et al. (2), who concluded that, in the Italian population, female longevity is more related to lifestyle and environmental conditions.

In the study of Young et al. (32), the levels of IL-6 from blood donors were analyzed using the automated Immulite assay and ELISA. They found different results in each of the techniques. The assay showed that men had higher IL-6 values in the 30–39 age group. In the older age groups, there was a reduction in IL-6 levels. They also found increased IL-6 levels in women in the 40–49 age group. When the data was analyzed using ELISA, women had higher levels of IL-6 in the 60–69 age group, but no differences were found between genders (32). In our study, even though it was possible to identify that changes in the IL-6 levels occurred at different stages in men and women, only the 51–60 age group showed significant differences between males and females.

Regarding hsCRP, the 51–60 age group had the highest values. However, when we analyzed this marker as a function of age, a positive correlation was found, i.e., increased levels of hsCRP with aging. This finding concurs with other studies in the literature (33). According to one study, because CRP is a nonspecific marker of inflammation (34), it can suffer the influence of a number of factors, including obesity, hypertension, smoking, increased levels of triglycerides, and others (35). Meanwhile, some studies indicate that CRP levels are associated with dietary patterns (36). In the present study, blood sampling was collected after 12 h of fasting, therefore all subjects were in the same dietary status. In addition, other variables that can alter the levels of CRP, such as obesity and smoking, were exclusion criteria for the study. Furthermore, statistical analyses were performed to ensure that the levels of triglycerides and LDL were not influencing the results.

As previously mentioned, positive correlations between inflammatory markers and age were found in the overall data (110 participants) and in the data divided by gender (male and female); however, women showed stronger correlations because younger women had lower values for inflammatory markers and older women had higher values, albeit non-significant, compared to men. This finding contradicts the study by Young et al. (32), who only found a positive correlation between IL-6 and age in males. Nevertheless, there are studies that also identified a positive correlation in both genders. Straub et al. (37) studied the levels of IL-6 in 120 subjects divided by gender and found a correlation of 0.41 for men and 0.48 for women, but unlike our study, the age of the subjects ranged from 15 to 80 years. These results need to be investigated further, particularly with respect to dividing data by gender. The conflicting findings are probably due to differences in methods of analysis, the sample sizes studied, and difficulty in selecting healthy subjects (32).

## Conclusion

In conclusion, the natural aging process caused increased levels of IL-6 and hsCRP, which is consistent with the theory proposed by inflammaging. Women presented stronger correlations compared to men for both IL-6 and hsCRP, and the 51–60 age group seemed to be a key point for the increase in these variables. Our findings are important because they indicate that preventive measures in earlier stages of life can minimize the increase in this inflammatory marker in natural aging.
